# New Urbanization and Rural Tourism Development under the Rural Revitalization Strategy Environment

**DOI:** 10.1155/2022/4095446

**Published:** 2022-08-21

**Authors:** Lujuan Jiang, Leilei Wang

**Affiliations:** ^1^College of History Culture and Tourism, Guangxi Normal University for Nationalities, Chongzuo 532200, China; ^2^College of Architecture and Landscape, Universiti Teknologi Malaysia, Skudai, Johor Bahru 81310, Johor, Malaysia

## Abstract

China can effectively promote urban-rural integration and economic and social modernization through new urbanization, which also serves as a strong driver and supporter of the growth of rural tourism. This paper examines the new urbanization and the growth of the rural tourism industry based on the rural revitalization strategy. It does so by using the techniques of literature research, field investigation, information technology retrieval, and excavation. We list the accomplishments of the rural tourism sector at its current stage of development and identify the issues and factors that will affect the sector's future growth. In addition, a coordinated development evaluation index system is built based on a theoretical analysis of rural revitalization strategies and new urbanization, and the corresponding comprehensive score is obtained using the entropy method for research. The index weight of the subsystem for rural revitalization in province A is computed using the entropy weight method. According to the findings, the wealth of life has the smallest weight (0.1117), followed by the prosperity of industry (0.2618), which is the largest on a criterion level. The effective weight of governance is the largest, at 0.2801. This study can serve as a useful resource for fostering rural tourism and advancing rural business.

## 1. Introduction

The rapid urbanization that has occurred in recent years contrasts sharply with the rapid rural decline [1]. On the one hand, a lot of rural talent moves to urban areas, which overly concentrates and saturates the urban talent pool. On the other hand, rural areas experience low income, subpar infrastructure, and a significant exodus of talent, particularly skilled talent. On the contrary, as new urbanization is encouraged and urban and rural development is better coordinated, the area of urban land is constantly growing, radiating to the surrounding areas, encroaching on excellent rural farmland, and seriously harming the rural ecological environment [2]. All three levels of the proposal—strategic level, institutional level, and rural revitalization strategy—presented fresh subjects and directions for further study in rural planning. Looking back at the aforementioned turning points in history, the nation made prodigious strides in rural development every time it modified and optimized its rural policies. We think that as reforms progress, rural development will inevitably make the transition from providing enough food and clothing to realizing the dream of leading a rich life, and the rural revitalization strategy offers the chance to do so [3]. By allocating resources as efficiently as possible, new urbanization will support the growth of rural revitalization. The growth of new urbanization will encourage the free flow of resources in towns and cities, as well as the maximum participation of all types of production factors that influence economic development [4]. The limitations of the city are gone, and the countryside can now access more materials and resources to advance more quickly and effectively and achieve rural revitalization.

How to rationally utilize distinctive regional characteristics and cultural connotations in the process of new urbanization to foster the development of a people-oriented local economy, realize the citizenization of agricultural migrants, maximize their layout and form, make them sustainable, and encourage the integration of urban and rural areas is a challenge that merits careful consideration and research [5]. Urban residents have a demand for environmentally friendly leisure travel in the suburbs due to the economy's rapid growth and the notable improvement in living standards [6]. Rural tourism can successfully meet this demand. Rural tourism will also encourage the exchange of resources between the urban and rural areas and the growth of ancillary industries like catering, sightseeing, agricultural product trading, hands-on farming experiences, agricultural culture and education, and parking lot management. However, there are many issues with rural planning, including a flawed planning management system, various planning unit levels, a lack of rural planning talent, an unreliable method for assessing the success of rural planning initiatives, and inadequate development of rural planning characteristics [7]. Based on this, this paper investigates how high-level rural planning and construction support rural revitalization strategy and how to use planning techniques to prevent issues that currently exist in rural development.

The tourism sector is one of the most powerful forces for development during the process of new urbanization. Its regionality defines the distinction between the tourism industry and the cultural industry, which will unavoidably increase the competitiveness of the integrated development of the cultural tourism industry and cause it to grow continuously, which will feed back on the growth of new urbanization, and the three will promote one another and grow together. We develop rural tourism, create a system for the rural tourism industry that demonstrates regional traits, embodies rural values, captures the essence of rural life, and adapts to modern needs, and encourage the growth of rural industry. The innovations of this paper are as follows:

1. Based on the background of rural revitalization strategy, this paper discusses the problems of new urbanization and rural tourism development. It is of great significance to explore the new path of new urbanization development in the new era, and the innovative development of tourism industry is an exploratory path. Therefore, this research is a fundamental and contemporary issue in both theory and practice, and it is closely linked with reality, which has important practical significance.
2. Developing rural tourism vigorously, scientifically directing rural urbanization, and encouraging the interactive and coordinated development of urban and rural tourism are crucial research areas for China's new urbanization and creation of stunning rural areas. In this study, the index system for measuring the degree of rural revitalization is built, and the entropy method is used to calculate the overall score. Based on the calculation of the coupling coordination degree, we further investigate the driving forces that influence the level of coordinated development of rural revitalization and new urbanization, and offer theoretical support for the coordinated development of the two.

## 2. Related Work

Lai et al. pointed out that only by transferring a large amount of surplus rural labor to employment in nonagricultural industries and completing the transition from rural residents to urban residents can the level of land scale management per household in rural areas be greatly improved; agricultural modernization will gradually create conditions [8, 9]. Zhou et al. pointed out that in order to successfully achieve the goals of the rural revitalization strategy, it is necessary to coordinate the relationship between the new urbanization strategy and the rural revitalization strategy, use the urban economy to fed back and drive the rural economy, and use the urbanization strategy to boost the rural revitalization strategy. Mutual cooperation with the market realizes a win-win situation between urban and rural interests, social public interests, and the interests of market players [10]. Abdollahzadeh et al. believed that in the process of urbanization, urbanized land use has an adverse impact on the development of rural tourism in suburban areas. Urbanized land will destroy the rural settlement landscape in suburban areas and is not conducive to the development of rural tourism in suburban areas [11]. Ikechukwu et al. established the evaluation index system of urban-rural integration development from the perspectives of space, economy, society, and ecological environment from the perspective of rural revitalization. The development level of urban-rural integration in a certain region is analyzed by using the analytic hierarchy process [12, 13]. On the premise of verifying the spatial correlation, Sikora et al. constructed a spatial Dubin space-time double-fixed model to explore the driving factors affecting rural revitalization and new urbanization [14]. The results of the model show that the level of location traffic, income driving, and equalization of public services in adjacent areas have a positive impact on the degree of coupling and coordination between the two in this area. The two coupling coordination degrees are negatively correlated. Gao et al. summarized and explored the problems existing in the current rural planning, and then carried out countermeasure research and analysis based on the problems; finally, we combined with the current situation of rural planning and construction in a certain place, and the research results were applied to the practical research of rural planning. The problems and applicable countermeasures in the planning are studied and analyzed [15]. Jepson et al. believed that the development of rural tourism is based on rural resources, and rural tourism is one of the new tourism modes of tourism [16]. Jasinskas et al. pointed out that rural industrial integration is the application and innovation of industrial integration theory in rural economic development integration [17].

This paper uses data mining technology to investigate the development of rural tourism and new urbanization under the rural revitalization strategy, based on a thorough discussion of prior literature. The index system of rural revitalization level is constructed in this paper, and the comprehensive score is obtained using the entropy method. Theoretical justification for the coordinated development of rural revitalization and new urbanization is provided on the basis of further exploration of the driving factors that affect the coordinated development level of the two. The results of the analysis are also visually presented at the same time thanks to computer technology. We study the rural tourism of the happy farmhouse's temporal and spatial distribution law, high-frequency vocabulary in the network platform, and hot topics in rural tourism. This study can serve as a resource for enhancing rural industries and growing rural tourism.

## 3. Methodology

### 3.1. Coordinated Development between Rural Revitalization and New Urbanization

Instead of being isolated, independent, and developing differently, it should be coordinated with the urban and rural areas. The advantages and characteristics of rural areas must be maintained, and urban and rural areas should complement one another. The countryside must also be the focus of current development to create a more harmonious whole. This is in line with the urbanization of the economy, population, environment, society, and rural areas [18]. In order to better implement the rural revitalization strategy, it is important to focus on rural planning, scientific planning, and rational spatial layout, as well as overall consideration of the development and planning of population, culture, medical and health care, society, economy, and road infrastructure at the township level. Additionally, it is important to further optimize the ecological spatial layout of production and living at the township level and to promote integration and diversity. Urbanization levels can vary depending on a number of factors, including the process by which traditional agricultural production and lifestyle are changed into new production modes, as well as the alteration of values, learning styles, thoughts, and emotions. New urbanization and rural revitalization are two opposing systems that collide and interact. The prosperity of rural industry can provide a large number of raw materials and basic factors of production for economic and social development. The prosperity of the rural industry will certainly make a large number of rural labor force turn to the industrial market, and this part of the demographic dividend will contribute to China's economic and social construction. The schematic diagram of the integration of new urbanization and cultural tourism industry is shown in Figure 1.

Rural tourism can be characterized as a specific type of tourism activity with its primary target market being urban residents and its main selling points being the rural natural environment, rural scenery, rural culture, agricultural production, and peasant life. In China, rural revitalization is being pushed forward by the combination of rural tourism and new urbanization, which has the potential to significantly advance the rural economy [19]. Villages and towns, which are the new urbanization's target areas, offer room, transportation, and platforms for the development of the industrial sector. The development of new urbanization has the potential to shift the surplus labor force to the industrial construction sector, separating the labor force in rural areas from the previous agricultural production in those areas. This not only helps to improve the income level of rural population but also forces the development of agricultural industry to a certain extent, because the decrease of agricultural population forces the agricultural production efficiency to be improved. The increase of income level has brought rural residents closer to a rich life. The development of rural tourism industry contributes to the local urbanization of rural areas and promotes the integration of urban and rural areas. Rural tourism brings abundant tourists to rural areas, satisfies the extension and development of industrial chain in rural areas, increases residents' income in rural areas, and promotes the realization of the goal of overall planning between urban and rural areas. The ultimate goal of rural revitalization is to achieve the growth that people yearn for a better life and to really improve farmers' sense of acquisition and happiness [20].

Because new urbanization adheres to people-oriented and ecological livability, building ecological villages and towns has grown in importance as a result. Doing so necessitates undertaking greening and beautification projects, reducing pollution from production and daily life, and raising the bar for environmental quality. Building ecological villages and towns has the potential not only to improve the rural environment but also to foster the growth of rural tourism by creating a beautiful rural ecological environment. This is known as the ecological coupling between rural tourism and villages and towns. This essay chooses a relevant urban population situation where there has been an increase in recent decades. From 2009 to 2019, Figure 2 depicts China's urbanization rate and the urbanization rate of the registered population.

On the whole, the urbanization level of China's population is on the rise, but the growth rate has slowed down in some years.

Urban development is currently far ahead of rural areas, and the dual development mechanism of urban and rural areas also has many drawbacks, which are the main issues in the coordinated development of urban and rural areas. The strategy of rural revitalization is a crucial first step in the development of rural areas, according to assessments of the state of urban and rural development and a thorough understanding of foreign countries' experiences. The tertiary sector of the Chinese economy, which has a significant positive impact on economic growth, includes tourism. It is the heart of cultural tourism, and travel is how culture is transported and developed. As a result of their close ties and interdependence, as well as the fact that they share many traits and qualities, the industries of industry and tourism are mutually beneficial and coprosperous. The blending of culture and tourism has emerged as a significant trend. Rural residents can improve their ideological quality, learn more about tourists' lifestyles and ideas, and alter their behavior and hygiene practices through contact with tourists. The challenges faced in developing the rural tourism industry are not only personal problems for individuals but also public social problems because it is one of the efficient ways to realize the prosperity of the rural industry and contributes positively to achieving the strategic goal of rural revitalization. Therefore, the management of issues facing the rural tourism sector falls under the purview of public governance [21]. As the most powerful force behind new urbanization, tourism is crucial to the process. Its regionality determines the differences, which will undoubtedly increase the competitiveness of the integrated development of the cultural tourism industry and encourage continuous growth. Although coupling and collaboration both represent the process of mutual influence between many systems, that is, from chaos to order, from low level to high level, the coupling will typically be interfered by external factors, and the corresponding collaboration is more represented as the process of internal influence between systems. It is possible to realize the collision of cultural exchanges and the effective utilization of rural resources through the integration and development of new urbanization and rural tourism, thus realizing the social and cultural coupling between them.

### 3.2. Data Mining and Analysis of Rural Tourism in the Era of Big Data

The distinctive qualities of new urbanization-urban-rural integration and urban-rural integration are intimately connected to the tourism sector. With the adjustment of the rural industrial structure, the needs of wealthy farmers, and the leisure travel of urban residents, rural tourism has emerged as a new driver of the tourism industry's growth. Numerous platforms have produced hundreds of millions of pieces of data about rural tourism as a result of advancements in communication technology, the growth of new media and social networks, and the arrival of the big data era. The tourism industry is currently facing a serious challenge regarding how to mine, process, and analyze big tourism data. The ultimate goal of data mining is to discover and deduce valuable knowledge, including concepts, rules, patterns, and models, and provide reference and support for management and decision making. This technology integrates the theories and technologies of mathematical statistics, database technology, machine learning, artificial intelligence, neural network, computing technology, visualization technology, and other fields. It is the sublimation of data from perceptual knowledge to rational knowledge. We can analyze and mine the data of “rural tourism” through various platforms for publishing information. The data mining architecture is shown in Figure 3.

The emphasis shift from the development of people to the scale expansion of urban construction, the emphasis on the citizenization of rural populations, the promotion of social equity, the overall planning of urban and rural areas, and the enhancement of the quality of urbanization in China are the main components of the transformation from urbanization to new urbanization. The fusion of rural tourism with new urbanization can foster the growth of three key industries, satisfy the demand of urban residents for rural tourist destinations, and foster the growth of regional rural-related industries. It can increase the revenue of the service sector in rural tourist destinations, lessen the seasonal economic disjointed impact of farming production in rural areas during lean farming, and revitalize rural economic development. We can see from the fundamental components of the new urbanization strategy and the rural revitalization strategy that both are based on the objective of the sustainable development of the entire Chinese society. The goal of this paper is to set up an index system to investigate the degree of coordination between new urbanization and rural revitalization in various provinces and cities. Therefore, we should choose an index that can capture the distinctions between urban and rural areas, compare those distinctions, and identify any potential remedial measures. This paper develops a new index system of urbanization and rural tourism development based on the principles of scientificity, systematicness, guidance, guidance, data availability, dynamics, and independence.  Table 1 displays the index system that was developed in this paper.

This paper uses the thorough index approach. Changes in space, economy, and population are all a result of the new urbanization. Planning for both urban and rural areas, economic and intensive development, livable environments, and a focus on people are the fundamental traits of new urbanization. The new urbanization begins with the fundamental issues, adheres to the principle of basing itself on national conditions and adapting to local conditions, and fundamentally departs from the previous conception of urbanization, which placed more emphasis on people than on other people. It aims to improve agricultural migrants' ability and quality, as well as their ability to participate equally in society and to develop on an equal footing, as part of the process of promoting migrant workers' citizenization.

Considering that some indicators are positive indicators, the larger the value, the stronger the positive effect on the comprehensive index. Some indicators are negative indicators. The smaller the value, the stronger the positive effect on the composite index. Therefore, this paper adopts the following standardization methods:

(1) $$\begin{array}{c} u_{ij}=\frac{x_{ij}-\min\left(x_{ij}\right)}{\max\left(x_{ij}\right)-\min\left(x_{ij}\right)},\\ u_{ij}=\frac{\max\left(x_{ij}\right)-x_{ij}}{\max\left(x_{ij}\right)-\min\left(x_{ij}\right)},\\ i=1,2,3,\ldots ,m\;j=1,2,3,\ldots ,n, \end{array}$$

where *u*_*ij*_ is the standardized processing result of the *j* th evaluation index in the *i* th comprehensive index; *x*_*ij*_ is the original value of the *j* th evaluation index in the *i* th comprehensive index; max(*x*_*ij*_) and min(*x*_*ij*_) represent the maximum value of the original value and the minimum value; *n* represents the total number of evaluation indicators in the comprehensive index; and *m* represents the total number of the comprehensive index.

To transform the proportion of indicators, the formula is as follows:

(2) $$\begin{array}{c} p_{ij}=\frac{x_{ij}^{\prime }}{\sum_{i=1}^{n}x_{ij}^{\prime }}. \end{array}$$

The specific calculation steps of the entropy value *A*_*j*_ of the data index of item *j* are as follows:

(3) $$\begin{array}{c} A_{j}=-k\sum_{i=1}^{n}p_{ij}\ln_{ij},\\ k=\frac{1}{\ln\left(n\right)},\\ k>0,\\ A_{j}\geq 0. \end{array}$$

We calculate the degree of difference of the first *j* indicator:

(4) $$\begin{array}{c} d_{j}=1-A_{j}. \end{array}$$

The comprehensive evaluation value *T*_*i*_ formula is as follows:

(5) $$\begin{array}{c} T_{i}=\sum_{j=1}^{m}w_{j}p_{ij}. \end{array}$$

In order to avoid the influence of missing indicators on the authenticity of the conclusion, the coefficient of variation method is used to deal with it. The specific formula is as follows:

(6) $$\begin{array}{c} v_{ij}=\frac{\sigma_{ij}}{\bar{x_{ij}}}. \end{array}$$

Among them, *v*_*ij*_, *σ*_*ij*_, and $\bar{x_{ij}}$, respectively, represent the coefficient of variation, standard deviation, and mean of the *j* th evaluation index in the *i* th comprehensive index, and the formula for calculating the weight of the *j* th evaluation index in the *i* th comprehensive index is as follows:

(7) $$\begin{array}{c} w_{ij}=\frac{v_{ij}}{\sum_{j=1}^{n}v_{ij}},\\ \sum_{j=1}^{n}w_{ij}=1. \end{array}$$

According to the characteristics of this research content and the above coupling relationship calculation model, the coupling degree model of rural tourism and new urbanization in this paper is designed as follows:

(8) $$\begin{array}{c} C={\left[\frac{\left(T_{1}\times T_{2}\right)}{\left(T_{1}+T_{2}\right)\times \left(T_{1}+T_{2}\right)}\right]}^{1/2}. \end{array}$$

In the formula, *T*_1_ is the value of rural tourism, and *T*_2_ is the value of new urbanization. The value interval of coupling degree *C* is [0, −1]. The larger the value, the greater the coupling degree and the higher the interaction between the two; that is, the better the coordination between rural tourism and new urbanization.

## 4. Result Analysis and Discussion

This paper chooses 20 provinces and cities in China as research objects, and further quantitatively analyzes the coupling coordination degree of rural revitalization and new urbanization in 20 provinces and cities from 2009 to 2019. This analysis aims to fully reflect the coordinated development level of rural revitalization and new urbanization, taking into account the availability of data. The degree of coordination is introduced to the coupling degree model in order to account for the degree of coordinated development of rural tourism and new urbanization, which the coupling degree model is unable to fully explain, as shown in Table 2.

At present, the development stage of China's tourism industry is basically consistent with the second stage of China's new urbanization process. Therefore, the integration of the two is not a unilateral reason, but a joint decision of their development. Integration is the inevitable result of new urbanization and the development of cultural tourism industry.  Figure 4 shows China's living affluence level from 2009 to 2019.

Generally speaking, although there is a gap between rural residents and urban residents, the level of living affluence of rural residents is still improving, and there is a tendency to narrow the gap between urban and rural areas. It can shape the unique and beautiful rural scenery in the countryside and take it as the core attraction to promote the development of rural tourism industry and optimize the rural industrial structure. To achieve industrial integration and development, we have embarked on a road of developing rural tourism industry to achieve rural industry prosperity. According to the entropy weight method, this paper calculates the index weight of rural revitalization subsystem in A province, and the results are shown in Table 3.

The results show that in terms of criterion level, the effective weight of governance is the largest, which is 0.2801, followed by the prosperity of industry, which is 0.2618, and the wealth of life is the smallest, which is 0.1117. Based on Sina Weibo in this chapter, through the analysis and exploration of rural tourism-related Weibo in A province, the analysis results are displayed visually. The average distribution of monthly index of relevant Weibo releases in 2010–2018 is shown in Figure 5.

In this paper, based on the Weibo data platform, we search for specific keywords, collect data, and analyze these data in depth to get the corresponding results.  Figure 6 shows the distribution of Weibo release time periods in a week.

The captured Weibo text content of “Farmhouse Rural Tourism” in province A is segmented.  Table 4 lists the top 30 high-frequency words and their corresponding word frequencies in the segmentation results.

According to the findings, the majority of farmhouse music-related rural tourism products in a province are rural restaurants and fruit and flower picking in the suburbs of the city. Local agricultural and sideline products are also used to draw tourists. This demonstrates that the level of farmhouse tourism products in the suburbs of province A is relatively low, that product homogenization is severe, and that seasonality is strong, all of which are detrimental to the market's long-term growth in rural areas. More data support is required for rural tourism, and the data should be thoroughly mined. Additionally, the government needs to pay attention to it, support it financially and in terms of building infrastructure, and direct and encourage the growth of the farmhouse music rural tourism market nationwide.

## 5. Conclusions

The natural ecology of the countryside should be preserved as we create a rural ecological civilization system and reshape the rural landscape for the postindustrial era. The development of rural areas will be encouraged to some extent by the creation of new industries, the revaluation of green mountains as assets, and the growth of distinctive tourism. In this study, the index system for measuring the degree of rural revitalization is built, and the entropy method is used to calculate the overall score. Based on the calculation of the coupling coordination degree, further investigate the driving forces that influence the level of coordinated development of rural revitalization and new urbanization, and offer theoretical support for the coordinated development of the two. The analysis results are presented visually at the same time thanks to computer technology. We examine the high-frequency words used on the network platform, the temporal and spatial distribution law of rural tourism of the happy farmhouse, and the current hot topics in rural tourism. According to the findings, the wealth of life has the smallest weight (0.1117), followed by the prosperity of industry (0.2618), which is the largest on a criterion level. The effective weight of governance is the largest, at 0.2801. This paper is intended to offer some theoretical research ideas and technical support for new urbanization and rural tourism development under the general guidelines of the new era's rural revitalization strategy. However, there are some restrictions in this paper's evaluation system and method for determining index weights. More adaptable techniques and metrics will be chosen in the future as one of the research trajectories.

## Figures and Tables

**Figure 1:** Schematic diagram of the integration of new urbanization and cultural tourism industry.

**Figure 2:** Urbanization rate and urbanization rate of registered population in China from 2009 to 2019.

**Figure 3:** Data mining architecture.

**Figure 4:** Living affluence level in China in 2009 to 2019.

**Figure 5:** Average distribution of monthly index of relevant Weibo releases in 2009 to 2019.

**Figure 6:** Distribution of Weibo release time period in a week.

**Table 1:** Index system of rural revitalization level.

Target layer	Criteria layer	Index layer	Unit	Attribute
Rural vitalization	Industrial prosperity	Agriculture accounts for total output value	%	Positive index
		Total mechanical power per unit sown area	KWh/ha	Positive index
		Grain yield per unit area	Tons/ha	Positive index
	Ecologically livable	Sanitary toilet penetration rate	Ten thousand kwh	Positive index
		Application amount of agricultural chemical fertilizer per unit sown area	Tons/ha	Negative index
		Number of hospital beds per 10,000 people in township	PCs/10000 persons	Positive index
	Affluent life	Per capita disposable income of rural residents	Yuan/person	Positive index
		Number of mobile phones per 100 rural households	PCs/100 households	Positive index
		Rural Engel index	%	Negative index
	Effective governance	Gini coefficient of farmers	%	Positive index
		Proportion of expenditure on urban and rural affairs in fiscal expenditure	%	Positive index
	Rural civilization	Township cultural station	Number	Positive index
		Rural residents' per capita expenditure on education and culture accounts for the total expenditure.	%	Positive index
		Average years of education of farmers	Year	Positive index

**Table 2:** Grading standard of coupling coordination degree.

Coordination level	Coupling degree interval	Coordination state
1	0.10–0.20	Serious maladjustment
2	0.20–0.30	Moderate disorder
3	0.30–0.40	Mild disorder
4	0.40–0.50	On the verge of maladjustment
5	0.50–0.60	Reluctantly coordinate
6	0.60–0.70	Primary coordination
7	0.70–0.80	Moderate coordination
8	0.80–0.90	Good coordination
9	0.90–1.00	Quality coordination

**Table 3:** Indicator weights of rural revitalization subsystem in province A.

Target layer	Criteria layer	Weight	Index layer	Unit	Attribute	Weight
Rural vitalization	Industrial prosperity	0.2618	Agriculture accounts for total output value	%	Positive index	0.0625
			Total mechanical power per unit sown area	KWh/ha	Positive index	0.0802
			Grain yield per unit area	Tons/ha	Positive index	0.0618
	Ecologically livable	0.1924	Sanitary toilet penetration rate	Ten thousand kwh	Positive index	0.0312
			Application amount of agricultural chemical fertilizer per unit sown area	Tons/ha	Negative index	0.0251
			Number of hospital beds per 10,000 people in township	PCs/10000 persons	Positive index	0.0132
	Affluent life	0.1029	Per capita disposable income of rural residents	Yuan/person	Positive index	0.0786
			Number of mobile phones per 100 rural households	PCs/100 households	Positive index	0.0197
			Rural Engel index	%	Negative index	0.0089
	Effective governance	0.2815	Gini coefficient of farmers	%	Positive index	0.0302
			Proportion of expenditure on urban and rural affairs in fiscal expenditure	%	Positive index	0.0904
	Rural civilization	0.1794	Township cultural station	Number	Positive index	0.1098
			Rural residents' per capita expenditure on education and culture accounts for the total expenditure.	%	Positive index	0.0351
			Average years of education of farmers	Year	Positive index	0.0254

**Table 4:** High-frequency words and corresponding word frequencies.

Keyword	Word frequency	Keyword	Word frequency
Eat	1846	Play	603
Travel	1803	Activity	598
Village	1724	Take stock of	592
Good	1706	Can	586
Travel	1588	Friend	571
Hill	1274	Today	549
Household	1021	Lake	536
Have leisure	948	Ecology	524
Be self-drive	903	Blow	519
Delicacy	854	Pluck	495
Vegetable	806	Pond	451
Countryside	702	Town	443
Weekend	694	Lotus	428
Suit	652	Be free of charge	419
Hamlet	614	Mature	408

## Data Availability

The data used to support the findings of this study are available from the corresponding author upon request.
